# PCNL Combined with 3D Printing Technology for the Treatment of Complex Staghorn Kidney Stones

**DOI:** 10.1155/2022/7554673

**Published:** 2022-03-15

**Authors:** Yubao Liu, Haifeng Song, Bo Xiao, Weiguo Hu, Gang Zhang, Meng Fu, Jianxing Li

**Affiliations:** Department of Urology, Beijing Tsinghua Changgung Hospital, School of Clinical Medicine, Tsinghua University, Beijing, China

## Abstract

**Objective:**

To explore the clinical application value of percutaneous nephrolithotripsy (PCNL) combined with 3D printing technology in the treatment of complex staghorn kidney stones.

**Methods:**

From January 2018 to February 2020, a total of 72 patients with complex staghorn kidney stones admitted to our center were divided into experimental group (3D printing group) and control group (computed tomography, CT, imaging group)) according to the random block method, and a prospective cohort study was conducted. Preoperative computed tomography urography (CTU) examination was performed on all patients in the two groups, and the original CT scan Digital Imaging and Communications in Medicine (DICOM) data of patients in the experimental group were separately extracted for three-dimensional reconstruction and 3D model printing and designed a doctor-patient communication evaluation score table. The two groups were compared in score table, puncture location time, total operation time, consistency between estimated calyx and target calyx, incidence of surgical complications, stone free rate, postoperative recovery, and other aspects.

**Results:**

Both groups completed preoperative CTU examination and showed good kidney and stone morphology. In the experimental group, all 3D printed models were completed and the internal anatomical structure could be clearly displayed. Simulation puncture and relevant measurement parameters could be obtained. The experimental group was significantly better than the control group in doctor-patient communication evaluation score, puncture location time, target calyx consistency, and stone free rate (*p* < 0.05), and there was no statistical difference in total operation time, postoperative complications, and postoperative recovery.

**Conclusions:**

Individualized 3D printing technology can fully evaluate and design percutaneous renal access and stone clearing strategies before surgery. Compared with traditional preoperative imaging evaluation, 3D printing makes PCNL more accurate and efficient in the treatment of complex staghorn shaped kidney stones, with a high stone free rate at the first stage and better doctor-patient communication satisfaction.

## 1. Introduction

PCNL characterized by small trauma and high stone-free rate has become the golden standard for the treatment of staghorn renal calculi, multiple renal calculi, or renal lower calyx calculi [1]. The risk of surgery and the stone-free rate are largely related to the selection and establishment of the percutaneous renal working tract. Therefore, it has become the key of PCNL surgery to confirm the relationship between the kidney and the stones, reasonably plan the renal target calyx to be chosen before surgery, and optimize the operational process of stone removal. At present, traditional kidney ureter bladder (KUB) and CT examinations cannot provide a comprehensive and detailed anatomical relationship between kidney stones and the collecting system, so it is difficult to obtain accurate preoperative evaluation and surgical design. 3D printing is a new rapid prototyping technology of advanced development in recent years. Based on the digital model file, it uses adhesive materials such as plastic and (or) powdered metal, turning blueprint on the computer into physical object through layer-by-layer printing according to computer aided design pattern [2, 3]. With continuous development of medical image technology and material engineering, 3D printing technology has been gradually extended and applied in medical practice. Compared with simple imageological diagnosis, the advantage of 3D printing is that doctors can print out a specific mould or organ model according to clinical needs and the individual difference of the patients' visceral organs, making it possible to diagnose more accurately and plan a detailed operation solution on printed physical models. Especially in department of orthopedics, plastic surgery, etc., have shown a huge clinical advantage. From January 2018 to February 2020, we made 3D models for 36 patients with staghorn kidney stones of our medical center, doing a preliminary study of surgery planning and the application of doctor-patient communication through 3D printing technology in PCNL.

## 2. Objects and Methods

### 2.1. General Information

From January 2018 to February 2020, we used random grouping method to divide 72 cases of PCNL patients into experimental group (3D printing group) and control group (CT imaging group). The treatment group included 36 cases four cases with hypertension disease and three cases with diabetes and one case underwent extracorporeal shock wave lithotripsy (ESWL) treatment 2 times. The control group included 36 cases five cases with hypertension and three with diabetes and three cases underwent ESWL treatment (one with 3 times and two with 2 times). The more preoperative demographic characteristics and specific parameters of two groups, such as age, gender, body mass index (BMI), stone size, and density (Hounsfield unit, HU), are shown in Table 1.

### 2.2. Production of 3D Models

#### 2.2.1. CT Examination

750HD 64 row CT (General Electric Company, GE) was used to obtain basic data. The renal CT data of the patients included the plain scan, arterial phase, venous phase, and excretory phase. During enhanced scanning, nonionic contrast agents were injected from anterior cubital artery with a dosage of 1.5∼2 ml/kg, a total of 80–100 ml, and an infusion speed of 2.0–2.5 ml/s. After the injection, continuous scanning was started in the four phases. The 5 mm thick image data layer was thinned to 1.25 mm and uploaded to the workstation.

#### 2.2.2. Image Postprocessing

The DICOM data files of the four phases were extracted and imported into mimics 19.0 3D image editing software for postprocessing. Specific steps: (1) Image segmentation: in order to extract objects for observation, the images were divided into several specific regions with unique features based on threshold segmentation, regional segmentation, etc. (2) The arterial stage model was set as the standard, the renal reconstructed model at the venous stage and excretory stage was introduced, and some characteristic markers were used for computer calculation and match. Then, conducted artificial auxiliary adjustments through three-dimensional *X*, *Y*, *Z* axis to match one by one, record coordinates, and achieve 3D images integration precisely. (3) Adjustment of the model: smoothing, denoising, filling, etc. The digital 3D model of the kidney was formed by rendering each structure value and adjusting transparency. Finally, the Standard Template Library (STL) format was output.

#### 2.2.3. 3D Model Printing

Object 260 printers from Stratasys company(USA) were used, workstation compatibility: Windows 7, 32/64 bit; size: 870 × 735 × 1200 mm. Print layer thickness: 16 microns; printing material: ① Vero material series: Tango series rubber flexible material, Veroclear, and RGD720 transparent material; ② digital materials: rigid opaque bright mixed materials and Shao A hardness value rubber materials; ③ support material: FullCure705 gel photosensitive polymer. Thermoplastic plastic is used for printing according to 3D reconstruction image in STL format. The renal parenchyma was soft transparent material, which is convenient for preoperative simulate puncture. After the 3D printing, the model was artificially colored: the renal arteries were red, the renal veins were blue, the renal collecting system and the ureter were yellow and milk white, and the kidney stones were rose red.

### 2.3. Preoperative Design and Surgical Methods

#### 2.3.1. Preoperative Design Planning

We used the 3D printing model as preoperative planning in experimental group while using CT imaging in control group. The two groups respectively design preoperative plan to decide targeting puncture renal calyx, tract number and sequence, stone clearing process, etc., and to measure and record related indexes such as the included angle, width, and length of the calyceal neck.

#### 2.3.2. Surgical Method

The operations of both groups were performed by the same young physician and assistant. Under general anesthesia and in the lithotomy position, a 5 French (Fr) ureteral catheter was inserted retrograde to the pelvis to perfuse the collecting system and prevent the stones falling down. Then, change to a prone position. According to the preoperative planning and design of the two groups, the target calyces were further confirmed by intraoperative ultrasound. A coaxial needle was introduced into the fornix of targeted calyx under ultrasound probe. The correct position was confirmed by aspiration of urine. A “J” shaped guide wire was passed through the needle into the calyces. After making a 1–1.5 cm incision, the tract was made step by step through the guide wire by the 8–16Fr fascial dilator (UroVision, Germany). The 16Fr peel-away sheath was left to facilitate the adjustment by ureteroscope (Storz, Germany). The working tract was dilated by 15–24Fr metal dilator to form a new 24Fr channel. The nephroscope (Richard Wolf, Germany) was placed into the collecting system through the tract and the stones were cleared by pneumatic lithotripsy and an ultrasonic system (EMS, Electro Medical System, Switzerland). At the end of the surgery, a 6Fr D-J stent was inserted antegrade into the ureter and 14Fr nephrostomy tube was placed. KUB reexamination 1–2 days after surgery was conducted to observe the location of D-J stent and significant residual stones.

### 2.4. Observation Index

#### 2.4.1. Preoperative

Doctor-patient communication evaluation score: ① preoperative communication time between doctor and patient; ② patients' cognition in 'disease (staghorn renal stone); ③ patients' understanding of surgical methods and risks; ④ patient's overall satisfaction. Among the ②–④ items, there are 5 grades with a total score of 100, which are good (90–100), relatively good (80–90), average (70–80), poor (60–70), and very poor (0–60). Patients are given scores according to their own understanding and communication.

#### 2.4.2. Intraoperative

(1) Puncture location time; (2) the consistency between the preoperative planned target calyx and the intraoperative actual target calyx; (3) total operation time.

#### 2.4.3. Postoperative

(1) Stone-free rate; (2) complications (bleeding, infection, organ damage, etc.); (3) postoperative recovery (postoperative recovery time and postoperative hospital stay).

### 2.5. Statistical Methods

Statistical analysis was performed using the SPSS for Windows version 19.0, the mean value was expressed using arithmetic mean and standard deviation, and measurement data used *x*±*s* to express. Chi-square and a 2-sample independent *t*-test were used. *p* < 0.05 was considered statistically significant.

## 3. Results

### 3.1. 3D Digital Image and Kidney Model

The 3D digital image of the stone-specific kidney reconstructed by DICOM data is clear and has good visual effect (Figures 1(a)–1(c)). 3D printed kidney models were able to present distinctly the renal vasculature, pelvis and calyx, ureter distribution, size, and location of the kidney stone. By simulating puncture and designing on the transparent renal parenchyma, good surgical effects were obtained (Figures 2(a)–2(d).

### 3.2. Observation and Evaluation Index

#### 3.2.1. Preoperative

3D printing model group showed obvious advantages in four aspects of doctor-patient communication evaluation score (Table 2). (2) Intraoperative: the 3D printing group was superior to the control group (*p* < 0.05) in two aspects: the puncture location time, the consistency between the preoperative planned target calyx, and the intraoperative actual target calyx. There was no significant difference in the total operation time (*p* > 0.05) between the two groups. (3) Postoperative: stone-free rate in 3D printing group is higher than that of the control group (*p* < 0.05). Postoperative complications: three cases in 3D printing group and two cases in control group were transiently bleeding in drainage tube postoperative 1–2 days and hemachrome changes within 3 g perioperative, and five patients accepted conservative treatment in stable condition. There were two cases in 3D printing group and two cases in control group accured postoperative fever. They were varying degrees urinary system infection cases indicated by preoperative urine routine test and urine culture, which continuously underwent antibiotic therapy. The body temperature of two patients in 3D printing group returned to normal about 3 days after receiving antibiotic treatment, and one patient in the control group recovered after 2 days, and the other patient did not improve significantly in 2 days, but returned to normal in 3 days after changing sensitive antibiotics. There were no blood transfusion, renal artery embolism, urinary sepsis, and peripheral organ injury in both groups. Postoperative recovery condition showed no significant difference between the two groups (*p* > 0.05) (Table 3).

## 4. Discussion

With the maturity of 3D reconstruction technology and image fusion, 3D engineering has been widely applied in medical industry such as orthopedics, stomatology, and plastic surgery, achieving initial effects [4–8]. Tansey [9] studied 20 cases of patients with hip fracture and evaluated the complex three-dimensional anatomical structure of the fractured pelvis and acetabulum through 3D print model, believing that the technology could help surgeons to understand the characteristics of complex fracture before operation and significantly reduced the interior variable degrees of fracture classification. Giovinco [10] applied 3D printing technology before the orthopedic surgery of Charcot foot syndrome to improve the probability of obtaining predictable surgical results and conducted preoperative simulation training which achieved good results. In the field of urology, Hulin Li [11] applied 3D reconstruction software to conduct image segmentation and 3D reconstruction and established a digital 3D model of renal calculi, which could clearly show the distribution of blood vessels in the patient's kidney and the spatial relationship between the renal collection system and the calculi. Yi Zhang [12] printed out 10 cases of models of kidney with tumor and applied them to preoperative planning of laparoscopic partial nephrectomy.

As for the diagnosis and treatment of complicated upper urinary tract calculi, especially in the treatment of staghorn calculi with PCNL, the operation is difficult and the learning curve is long. Currently, there is no relatively effective method to complete preoperative planning and simulation training; therefore, we tried to design preoperative planning guidance for PCNL using 3D printing technology. Most of the print models at present are solid or of achromatic color. For parenchyma organ, we have to observe the internal structure only by 3D digital image or disassembling the print model. In order to enhance the visual effect and improve the accuracy of preoperative design and patient cognition, we chose soft material to print transparent renal parenchyma through strengthening technologies successfully, because it was convenient for observation and simulate puncture. The collecting system, blood vessels, and stones were processed by selected color with high degree of distinction. The 3D model is 1 : 1 with the actual kidney.

As for the treatment of complicated renal stone with PCNL, it often requires multichannel or even multistage surgery, which greatly increases the risk of surgical bleeding [13]. Therefore, it is very important to design the puncture path, establish the passage, and make an overall plan of the stone removal steps before surgery. The routine preoperative KUB cannot reveal the structural characteristics of collecting system; moreover, the images of calculi in the pelvis and posterior calyx are generally overlapping, which confuses the determination of the puncture in the posterior calyx. CT scan has poor usage in the details and particular planning of overall stone removal. The 3D printing transparent model accomplished in this study clearly shows the three-dimensional shape of all internal structures for performers which allows observation and analysis from various angles. Renal parenchyma is printed with soft materials to facilitate the simulation of puncture in real time and the design of channel. The specific methods are as follows. At first, the posterior calyx has large stone with a wide and short calyceal neck which was taken as the first channel. The marking needle was used to puncture and locate through this renal calyceal fornix, and the marking needle was retained. Then, the anterior calyx paired with it or the adjacent calyx was found and punctured through the calyceal fornix with the marking needle. Then, the angle between the two needles was measured. If the angel was no less than 90°, generally, the nephroscope could enter the anterior or adjacent calyx from the posterior target calyx. That anterior or adjacent calyx would be defined as the first advantage calyx of the first channel in which stones were cleared first. If the angel was among 90° to 45°, the adjacent calyx would be defined as the second advantage calyx of the first channel. The selecting principle of the second channel is basically the same as that of the first channel. For staghorn calculi with more renal calyx and complex structure, this method is used in turn to design the working channels if more channels need to be established. The stones of the parallel calyx are individually marked. Finally, the planned punctured calyx and the sequence of stones clearance was recorded in detail.

Puncture location and stones clearance is based on accurate preoperative plan; surgeons can locate the target calyx more quickly and enhance the stone removal efficiency. This is the reason why the 3D printing group is superior to the control group in puncture location time and the stone free rate. However, the process of stone clearance, which accounted for a large proportion of the total operational time, largely depended on the stone composition and severity of renal obstruction, explaining why there was no significant difference in the total operation time of surgery between the two groups. The structure of the 3D model is completely consistent with the actual kidney, so the target renal calyx selected according to the model before surgery is basically consistent with the judgment of intraoperative ultrasonic position. For the control group, the target calyx selected according to CT evaluation before surgery can only serve as preliminary judgment, which needed to be assisted by actual intraoperative ultrasonic judgment. Therefore, there was a significant difference between the two groups in target calyx consistency. Surgical complications such as renal hemorrhage, urinary sepsis, and peripheral organ injury are related to the severity of urinary obstruction, stone size, operative experience, patients' obesity, and other conditions. In addition, the limited number of cases included in this study with adequate preoperative preparation and strict intraoperative operation also reduced the occurrence of surgical complications to a certain extent. Thus, there was no obvious difference between the two groups in postoperative complications.

During preoperative conversations with the patients and their family members, the surgeons took advantage of the visualized effect of 3D printing model to analyze and explain the renal structure, specific process of the operation, the possibility and reason of postoperative complications, making preoperative doctor-patient communication more rigorous and sufficient, promoted the patient to trust and obey the doctors, and raised the efficiency of conversation. The patients also believed it to be a good way of communication, and favorable results had been achieved. Patients' cognition of the disease and treatment may also be affected by a variety of other factors, such as educational background and previous history of PCNL surgery. Most of the cases included in this study had secondary education, and only two in the control group were undergraduates. There were a total of five cases (two in the experimental group and three in the control group) who had a previous history of PCNL surgery. Through preoperative conversation, it was learned that they only had a preliminary understanding of the operation, without in-depth perceive, and had not done any inquiry and research on it, so the bias of results caused by other confounding factors was basically excluded.

As 3D printing technology has not been widely reported in the diagnosis and treatment in the field of urinary calculi, the preliminary exploration and clinical application of this study provide part of the theoretical basis for preoperative planning of minimally invasive treatment of calculi. In the next stage of this research, it is planned to improve the microcontrol technology, making the relative space position between the third and fourth branch blood vessels, the calyces and stones more elaborate. Moreover, improve and refine the printing material, allowing the kidney model to clearly show the internal structure and stone images under ultrasound, making it possible for the performers and young physicians to do ultrasound-guided preoperative simulated puncture exercise, achieving the effect of simulated training as well as cultivating young physicians and shorten their learning curve.

At present, 3D printing technology is in the stage of preliminary exploration in the planning and designing of preoperative PCNL, and there are still some deficiencies. (1) Although the 3D printing technology can clearly display the main blood vessels of the kidney, it is still difficult to accurately print the blood vessels of third and fourth branch blood vessels. (2) In the preoperative simulated puncture process, the marking needle will leave deep needle trace in the renal parenchyma. As a result, repeated puncture will cause certain degree of disorder in the renal pelvis and renal calyx structure, which will affect the overall visual effect and interfere with the accuracy of the design program (3) Some cases had no hydrocalycosis and space so that these kidney models cannot be clearly distinguished but for color difference, resulting in the deviation of the operator's cognition. These problems will be further improved and solved in the follow-up research.

## 5. Conclusion

Our results supplement to the application of 3D printing technology in the field of urinary calculi, confirming the feasibility and effectiveness of preoperative planning and simulation of PCNL through 3D printed model of kidney with stones. It has certain clinical significance for precise design and reasonably planning operative steps as well as safely operating the surgery. 3D printing technology is an important step for digital virtual design to realize the transformation from virtual to reality, and it also has a promising prospect in the field of urology which means that technological innovation can better serve the patients.

## Figures and Tables

**Figure 1:** (a) 3D digital reconstruction of collection system and stones. (b) 3D digital reconstruction of collection system, stones, and vasculature. (c) Overall perspective of the 3D digital reconstruction.

**Figure 2:** 3D printing kidney model with stones. The renal arteries were red, the renal veins were blue, the renal collection systems were light yellow, the ureter was milk white and the stones were rose red. (a) 3D printing model of left kidney in ventral surface. (b) 3D printing model of left kidney in dorsal surface. (c) Simulating puncture in posterior upper calyx. (d) Simulating puncture in posterior middle calyx.

**Table 1:** The preoperative demographic characteristics of two groups.

Characteristics	3D printing group (*n* = 36)	CT imaging group (*n* = 36)	*p* value
Age (years)	45.1 ± 1.6	43.1 ± 2.1	0.438
*Gender*			
Male	19(52.7)	21(58.3)	0.422
Female	17(47.2)	15(41.6)	0.531
BMI (kg.m^−2^)	21.6 ± 1.2	22.9 ± 1.1	0.377
SCR (*μ*mol/L^−1^)	79.2 ± 2.1	81.2 ± 3.2	0.271
Stone size (cm)	6.8 ± 1.7	7.0 ± 1.4	0.227
CT values (HU)	1120 ± 130	1190 ± 220	0.121
Urine culture (+)	15	21	0.09
UTI	31	33	0.241

**Table 2:** Doctor-patient communication evaluation score.

Parameters	3D printing group (*n* = 36)	CT imaging group (*n* = 36)	*p* value
Communication time (mins)	12 ± 1.3	21 ± 2.1	0.018
Cognition in disease	92 ± 3.2	48 ± 2.1	0.009
Understanding in operation	96 ± 4.1	70 ± 3.1	0.011
Satisfaction	94 ± 3.2	81 ± 2.1	0.027

**Table 3:** Comparison between the two groups' intraoperative and postoperative observation index.

Parameters	3D printing group (*n* = 36)	CT imaging group (*n* = 36)	*p* value
Puncture location time (mins)	2.1 ± 0.8	3.5 ± 1.1	0.024
Target calyx consistency (%)	88.3 ± 6.2	61.4 ± 3.2	0.013
Tota1 operation time (mins)	112 ± 11.4	121 ± 21.5	0.315
Stone free rate (%)	83.1 ± 3.1	69.2 ± 3.2	0.014
Clavien Dindo < II complications	5	4	0.228
Postoperative recovery time (days)	2.3 ± 0.4	2.7 ± 0.2	0.121
Hospitalization time (days)	8.9 ± 1.1	9.3 ± 1.4	0.178

## Data Availability

The data used to support the findings of this study are available from the corresponding author upon request.
